# Three-Dimensional Ultrasound Imaging under Optimized Nuclear Regression Reconstruction Algorithm in the Diagnosis Vaginal Delivery and Cesarean Section on the Anal Sphincter Complex of Primiparas

**DOI:** 10.1155/2022/6173460

**Published:** 2022-06-07

**Authors:** Han Wang, Xiaolan He, Yi He

**Affiliations:** Department of Obstetrics and Gynecology, Wuhan First Hospital, Wuhan 430022, China

## Abstract

This study was aimed at analyzing the injury of anal sphincter (AS) for primipara caused by the vaginal delivery and cesarean section under the guidance of three-dimensional (3D) ultrasound images. A total of 160 patients who underwent postpartum reexamination were enrolled as the research subjects, including 80 cases of natural delivery (group A) and 80 cases of cesarean section pregnant women (group B), all of whom underwent three-dimensional ultrasound imaging scans. At the same time, an optimized kernel regression reconstruction (KRR) algorithm was proposed for the enhancement of ultrasound images. It was found that the running time after acceleration by the graphics processing unit (GPU) was obviously superior to that of a single-threaded CPU and a multithreaded CPU, showing statistical differences (*P* < 0.05). The thickness of the proximal and distal external AS in group A was much thinner in contrast to that in group B, showing statistical difference (*P* < 0.05). Therefore, the 3D ultrasound image based on the optimized KRR algorithm can accurately assess the morphology of AS injury in primipara, and the adverse effect of natural delivery on the AS complex in primipara was greater than that of cesarean section.

## 1. Introduction

In recent years, with the continuous progress and development of health awareness, women are paying more and more attention to their own health and recovery of postpartum pelvic floor function [1]. Anal sphincter complex (ASC) is the main component of the posterior pelvic cavity, and it is an important structure to maintain the normal exhaust and defecation of the anus. ASC is a morphological and functional unity composed of internal anal sphincter (AS), external AS, puborectalis, and combined longitudinal muscles. The delivery of pregnant women is the main cause of injury of ASC [2, 3]. The injury of ASC can cause fecal incontinence or exhaust incontinence, and the incidence can reach up to 60% [4]. Neurological or mechanical injury to the ASC caused by vaginal delivery is more common. For women who give birth in the vagina for the first time, about 30% of women will cause AS injury during the delivery process [5, 6]. A small number of pregnant women with cesarean section can also cause injury of AS. Studies have shown that about 2% of women who choose cesarean section will have symptoms of anal incontinence [7, 8].

At present, magnetic resonance imaging (MRI) and endoanal ultrasound (EAUS) are widely used in the diagnosis and evaluation of AS [9, 10]. With the continuous update and development of medical equipment, perineal ultrasound (translabial ultrasound (TLUS)) is increasingly used in the evaluation of female pelvic floor muscle function [11]. Compared with MRI, ultrasound diagnosis is cheaper, convenient, fast, and easier for patients to accept, and the diagnosis time is shorter, so it is more comfortable than rectal ultrasound diagnosis [12]. Although there are many advantages of 3D ultrasound, the speed of 3D ultrasound calculation is relatively slow, so the acceleration of its algorithm is a very critical step [13]. The freestyle 3D kernel regression reconstruction (KRR) algorithm is an algorithm that is very suitable for GPU acceleration, which can make the algorithm better put into practical use.

Compared with other algorithms, the KRR algorithm has better artifacts and higher graphics quality, but it also takes more time and cost to calculate [14]. The 3D ultrasound image reconstructed by the GPU-accelerated 3D ultrasound reconstruction algorithm can well reflect the shape of the original data volume, which can assist medical staff in diagnosis and effectively improve the efficiency of diagnosis and treatment. The KRR algorithm was constructed to accelerate the GPU, which can greatly reduce the running time of the algorithm for 3D reconstruction graphics. To sum up, the combination of artificial intelligence algorithm and imaging technology in clinical disease diagnosis is a hot research topic of scholars at present. In this study, 160 patients who underwent postpartum reexamination were included as the research objects, 80 cases of natural delivery were set as group A, and 80 pregnant women with cesarean section were set as group B, all of which underwent three-dimensional ultrasound imaging scans. At the same time, an optimized KRR algorithm was proposed to enhance the ultrasonic image processing, and then the changes of the anal sphincter complex in pregnant women under different delivery methods were comprehensively evaluated.

## 2. Materials and Methods

### 2.1. Research Objects

In this study, 160 cases of patients who were admitted to the hospital for postpartum reexamination from October 20, 2017 to October 20, 2019 were selected as the research objects, of which 80 cases were natural delivery (group A) and 80 cases were pregnant women with cesarean section (group B). The study had been approved by the ethics committee of the hospital, and the patients and their families signed the informed consent forms.

The inclusion criteria were defined as follows: primiparous women aged 20~30 years old; primiparous women whose singleton and third trimester ultrasound confirmed that the size of the fetus was in line with the gestational week, 42 days after delivery; the women undergoing cesarean section who were in the second stage; patients who had clear consciousness and were able to cooperate the study; and patients with no pelvic surgery.

The exclusion criteria were defined as follows: (1) patients with psychiatric diseases; (2) patients with incomplete clinical data; (3) patients who withdrew from the experiment due to their own reasons; (4) patients with speech and communication impairment, hearing impairment, or severe cognitive impairment; and (5) patients with psychiatric disorders.

### 2.2. Operation Methods

The ultrasonic diagnostic instrument was used to diagnose the patient. The ultrasonic probe frequency was 5-9 MHz intracavitary volume. The specific operation methods were defined as follows. The medical record number, age, height, delivery weight, fetal weight at birth, delivery method, and midwifery method of postpartum pregnant woman were recorded. The patient was instructed to take the lithotomy position ten minutes after defecation and urination, while flexing the hips and slightly abducting the knees. The female probe was coated with coupling agent and wrapped in a condom. The probe was placed at the patient's perineum to scan from bottom to top in the cross-section (from the end of the anus to the anorectal angle). The ASC was observed in multiple planes in the following three planes: proximal plane, middle plane, and distal plane. The thickness of AS inside the anus was measured at the 3, 6, 9, and 12 o'clock directions.

### 2.3. The Construction of Freestyle KR-Based 3D Ultrasound Reconstruction Algorithm

In the KRR algorithm of GPU version, the algorithm was divided into two parts: data acquisition and target reconstruction. The most important step was data acquisition, which directly affected the accuracy and efficiency of subsequent image reconstruction. Data acquisition was mainly completed by two parts. The first part was to calibrate the two-dimensional B-ultrasound image to determine its correct physical position; and the second part was to select the ultrasound observation area to be reconstructed. With the development of machine learning methods, the KRR algorithm began to be widely used. This idea was called the KR method in nonparametric estimation. The KRR-based 3D reconstruction algorithm was developed on this basis in this study.

After the initial filling stage, a discrete 3D ultrasound image data was obtained. Each point in this image can be expressed by equation (1) under nonparametric estimation:

(1) $$\begin{array}{c} A_{l}=f\left(Y_{l}\right)+\delta_{l},\text{l}=1,\cdots ,O, \end{array}$$

In the above equation (1), *A*_*l*_ referred to the observed value, *f*(.) was the regression equation, *Y*_*l*_ = (*Y*_*l*1_, *Y*_*l*2_, *Y*_*l*3_)^*n*^ was the 3D coordinates of the corresponding point, *δ*_*l*_ represented the noise error without interfere with each other, and 1, ⋯, *O* represented all the points in the 3D graph. If *Y*_*l*_ was a sampling point near the *Y* point, *f*(*Y*_*l*_) can be expressed as equation (2) below after incorporated with Taylor equation.

(2) $$\begin{array}{c} f\left(Y_{l}\right)\approx f\left(Y\right)+f^{\prime }\left(Y\right)\left(Y_{l}-Y\right)+\frac{1}{2}f^{\prime \prime }\left(Y\right){\left(Y_{l}-Y\right)}^{2}+\cdots \frac{1}{n}f^{n}\left(Y\right){\left(Y_{l}-Y\right)}^{n}. \end{array}$$

It could be transformed into

(3) $$\begin{array}{c} g_{0}+g_{1}\left(Y_{l}-Y\right)+g_{2}{\left(Y_{l}-Y\right)}^{2}+\cdots +g_{n}{\left(Y_{l}-Y\right)}^{n}. \end{array}$$

The above equation showed that if the Taylor function was considered the local performance of the regression function, then the estimated parameters *g*_0_ in the above equation can be expressed as the estimated solution of the regression equation when the data was *Y*_*l*_.

The regression equation obtained can reflect the real data only when *δ*_*l*_ closer to 0. The least squares equation was used to make the observed value *Y*_*l*_ closer to the value of the regression equation *f*(*Y*_*l*_):

(4) $$\begin{array}{c} \underset{\left(g_{n}\right)}{\min}\overset{o}{\underset{l=1}{\sum }}{\left[A_{l}-g_{0}-g_{1}\left(Y_{l}-Y\right)-g_{2}{\left(Y_{l}-Y\right)}^{2}-\cdots -g_{n}{\left(Y_{l}-Y\right)}^{n}\right]}^{2}\frac{1}{M}k\left(\frac{Y_{l}-Y}{M}\right). \end{array}$$

In the above equation, *k*(·) referred to the kernel function, and it was also a weighting function. It was mainly used to determine the influence of the points around the calculation point on the calculation point. If the surrounding points were farther from the calculation center point, the weighting effect would be worse, and the smoothing parameter *M* was used to control this influence. If the function was a symmetric function at this time, and its maximum value was 0, then it satisfied equation (5) below:

(5) $$\begin{array}{c} \int_{s^{1}}cj\left(w\right)ad=0,\int_{s^{1}}c^{2}j\left(w\right)ad=H. \end{array}$$

In the equation above, *H* was a constant value and *j*(·) was a Gaussian function. Just as the estimation shown in the least square method of the previous equation (4), parameter *M* affected the accuracy and complexity of the voxel in the local approximation. Therefore, the size of *M* was very important. The kernel function *j*(·) became a function with three directional variables, and its bandwidth *M* should be a 2∗3 matrix. The selected Gaussian function equation was as follows:

(6) $$\begin{array}{c} M^{-3}j\left(\frac{\left\|R\right\|}{M}\right). \end{array}$$

In equation (6), *M* was the bandwidth of the Gaussian function, and it was also the smoothing parameter introduced above. As a 3D point *X*, *Y* = (*Y*_1_, *Y*_2_, *Y*_3_)^*n*^ was found. For more convenient calculation, the *Y* value was set to 3. Based on the condition of 3D point, equation (4) could be equivalently transformed into the below equation:

(7) $$\begin{array}{c} \overset{0}{\underset{l=1}{\sum }}B_{l}\left(R\right){\left(A_{l}-g_{0}-\overset{3}{\underset{t=1}{\sum }}g_{t}\left(Y_{lt}-Y_{t}\right)\right)}^{2}, \end{array}$$

where *B*_*l*_(*R*) represented the impact of the point *Y*_*l*_ on the calculation point of the central point *Y*. The value was determined based on the distance from the point *Y*_*l*_ to the point *Y* and the corresponding bandwidth M, which could be expressed as follows:

(8) $$\begin{array}{c} B_{l}\left(R\right)=F\left(\frac{\left\|Y_{l}-Y\right\|}{M}\right). \end{array}$$

In order to facilitate the calculation of the computer, it had to solve the minimum case of equation (7) and convert it into the form of a matrix. For each point around the calculation point, there was a distance matrix *E*_*g*_ to store the distance from the surrounding points to the calculation point. The 3D matrix was shown as follows:

(9) $$\begin{array}{c} E_{g}=\left(\begin{array}{cccc} 1 & E_{11}-E_{1} & E_{12}-E_{2} & E_{13}-E_{3}\\ 1 & E_{21}-E_{1} & E_{22}-E_{1} & E_{23}-E_{1}\\ 1 & E_{31}-E_{1} & E_{32}-E_{1} & E_{33}-E_{1} \end{array}\right). \end{array}$$

This matrix was also the distance matrix that the CPU needed to prepare for GPU acceleration when the algorithm was implemented in the following algorithm. When the minimum value of equation (7) was obtained, the corresponding value of *λ*_0_, *λ*_1_, *λ*_2_, and *λ*_3_ was calculated with the below equation:

(10) $$\begin{array}{c} \overset{\wedge }{\lambda }={\left({\overset{\wedge }{\lambda }}_{0},\cdots ,{\overset{\wedge }{\lambda }}_{3}\right)}^{e}. \end{array}$$

It was assumed that the estimated value was $\overset{\wedge }{V}\left(E\right)$; the estimated value sought in this study was ${\overset{\wedge }{\lambda }}_{0}$ according to above descriptions. Thus, equation (11) could be obtained.

(11) $$\begin{array}{c} \overset{\wedge }{V}\left(E\right)={\overset{\wedge }{\lambda }}_{0}. \end{array}$$

After the distance matrix *E*_*g*_ was obtained, another matrix was needed to calculate the impact of the surrounding points to the calculation point, which referred to the distance weighting matrix. Obviously, the Gaussian function in equation (8) could be undertaken as a weighting reference. In consideration of the matrix form for finding the minimum of equation (7), a matrix *W*_*x*_ could be used, which was a diagonal matrix. The element value at (*x*, *x*) was *B*_*l*_(*R*) in equation (8). According to the above conditions, the matrix operation equation corresponding to the estimated value $\overset{\wedge }{V}\left(E\right)$ can be obtained as follows through matrix operation of equation (7):

(12) $$\begin{array}{c} \overset{\wedge }{V}\left(E\right)={\overset{\wedge }{\lambda }}_{0}=R_{1}^{i}{\left(E_{x}^{i}W_{x}E_{x}\right)}^{-1}E_{x}^{i}W_{x}Z. \end{array}$$

In the above equation (12), *R*_1_ was a column vector, only the first number was 1, and the others were all 0, aiming to find the solution of ${\overset{\wedge }{\lambda }}_{0}$ more convenient. *Z* was also a column vector, the pixel value corresponding to coordinate *E* was stored in the 3D ultrasound image, and the size of the vector was determined by *i*. However, since all points were not calculated in actual work, the calculation point was selected as the center, and a cube of size kSize∗kSize∗kSize was selected in the input of the 3D image, and the pixel value in the cube was taken as the value of *E*. The selection of kSize had a lot to do with the actual programming. The above all were the introductions of the 3D ultrasound reconstruction algorithm.

### 2.4. Statistical Methods

The data processing was analyzed by SPSS19.0 version statistical software. The measurement data was indicated as mean ± standard deviation ($\bar{x}\pm s$), and the count data was displayed as percentage (%). The running time was compared in pairwise using the one-way analysis of variance. The age, height, weight, course of disease, and diagnostic accuracy of patients between groups were compared with the paired *t* test. The difference was statistically significant at *P* < 0.05.

## 3. Results

### 3.1. Comparison on Basic Data of Patients

As shown in Figure 1, the average age of the patients in group A was 26.16 ± 3.98 years, the average height was 162.82 ± 5.09 cm, the average weight at delivery was 70.72 ± 5.81 kg, and the average weight of the newborn was 2.89 ± 1.02 kg. In group B, the average age, average height, average weight, average weight at delivery of the women, and average weight of the newborn were 27.19 ± 4.01 years, 159.73 ± 5.17 cm, 68.62 ± 6.71 kg, and 3.06 ± 1.12 kg, respectively. There was no statistical difference between the two groups of patients in the comparison of basic data (*P* > 0.05), so the experimental research can be carried out.

### 3.2. Comparison on GPU Acceleration Effect of KRR Algorithm

When the CPU acceleration effects were compared, the single-threaded CPU, multithreaded CPU, and GPU were selected, and the results were shown in Figure 2 below. The running time of single-threaded CPU was 17.62 ± 4.02 seconds, the running time of multithreaded CPU was 14.73 ± 3.07 seconds, and the running time of the GPU was 1.98 ± 0.03 seconds. Thus, the running time after GPU acceleration was more obvious, which was greatly different from the running time of single-threaded CPU and multithreaded CPU, showing meaningful differences (*P* < 0.05).

### 3.3. Comparison of the Calculation Parameters of KRR Algorithm to the Acceleration Effect

To analyze the impacts of different calculation parameters on the actual reconstruction effect, the different kSizes of the AS data with a size of 400∗289∗430 were selected for comparison, and the results were as follows. As illustrated in Figures 3–5, the size of kSize had a great influence on the computing time of the KR algorithm. When kSize = 6, the CPU computing time was 1372.52 ± 78.62 seconds, and when kSize = 8, the CPU computing time was 2478.56 ± 100.47 seconds, so the running time had increased by about 80%. When kSize = 10, the CPU computing time was 5583.17 ± 300.62 seconds, which doubled the time on the basis; in addition, the running time of GPU at kSize = 6 was 9.72 ± 0.07 seconds. When kSize = 8, the running time was 24.08 ± 1.03 seconds, and when kSize = 10, the running time was 50.02 ± 2.77 seconds. The running time had increased nearly twice. It indicated that the change of kSize could affect the reconstruction computing time of KRR algorithm, and the differences in computing time were obvious (*P* < 0.05).

Figures 6–8 showed the 3D tomographic images of AS of healthy people and the 3D ultrasound images of the patients after delivery. It showed that the structure of the perineum of healthy women was complete and the structure of the anal sphincter muscle was normal, while the structure of the perineum of the puerpera was incomplete, and the anal sphincter complex had a certain degree of rupture.

### 3.4. Comparison on as Measurement Results of Two Groups of Patients

Figure 9 illustrated that the thickness of the proximal external AS section measured at 12 o'clock and 6 o'clock was 1.42 ± 0.31 mm and 1.71 ± 0.37 mm, respectively, while those in group B were 1.83 ± 0.51 mm and 2.09 ± 0.43 mm, respectively. Thus, the AS in group A was thinner than that in group B, and the difference was remarkable in statistics (*P* < 0.05).

Figure 10 revealed that the thickness of the measured mid-extra-anal AS section at 12 o'clock was relatively weaker than that in group B, and the difference was obvious in statistics (*P* < 0.05).

In Figures 11 and 12, the measured thicknesses of the distal external AS section at 12 o'clock and 6 o'clock were 1.49 ± 0.33 mm and 2.14 ± 0.51 mm, respectively, while those in group B were 1.79 ± 0.62 mm and 1.97 ± 0.47 mm, respectively. The measured AS in the anus were 1.01 ± 0.021 mm and 2.88 ± 0.66 mm, respectively, and the AS thickness in group B were 1.94 ± 0.56 mm and 2.73 ± 0.52 mm, respectively. The thickness comparison between the two groups show huge difference (*P* < 0.05). The thickness of the puborectalis muscle of the two groups of patients was measured through experiments, and it was found that the thickness of both sides of the puborectalis muscle of the two groups did not change greatly (*P* > 0.05).

## 4. Discussion

ASC is an important part of maintaining anal self-regulation. Any part of ASC can cause anal defecation, gas incontinence, and other symptoms [15]. Therefore, accurate diagnosis and timely exercise and repair of injury of ASC are of great significance to reduce or avoid the occurrence of anal incontinence in the future [16]. The optimized freestyle KRR algorithm in this study had greatly improved the computational efficiency after GPU acceleration. The results showed that in terms of the CPU acceleration effect, the running time of single-threaded CPU was 17.62 ± 4.02 seconds, the running time of the multithreaded CPU was 14.73 ± 3.07 seconds, and the running time of GPU was 1.98 ± 0.03 seconds. The running time after GPU acceleration was the most obvious, showing dramatic difference (*P* < 0.05). The comparison of different kSize revealed that the size of kSize had a great impact on the computing time of the KRR algorithm. The running time of GPU was 9.72 ± 0.07 seconds when kSize = 6, 24.08 ± 1.03 seconds when kSize = 8, and 50.02 ± 2.77 seconds when kSize = 10. Such results indicated that the change of kSize could affect the reconstruction operation time of the KRR algorithm, and the operation time difference between them was large dramatically (*P* < 0.05). Such results suggested that the algorithm could be optimized to greatly increase the speed of calculation and can quickly make judgments for the diagnosis of the patient's condition, saving diagnosis time. This was more consistent with the research results of Wen et al. [17], and both show that the optimized KRR algorithm could not only improve the diagnosis effect but also shorten the calculation time and improve the overall diagnosis efficiency.

The optimized KRR algorithm was applied to the 3D ultrasound images of the primipara. It was found that the thickness of the measured proximal external AS section at 12 o'clock and 6 o'clock were 1.42 ± 0.31 mm and 1.71 ± 0.37 mm, respectively, while those in group B were 1.83 ± 0.51 mm and 2.09 ± 0.43 mm, respectively. The thickness of the measure AS section in group A was thinner than that in group B, with great difference (*P* < 0.05). This indicated that the anal sphincter complex was thinner in women who have given birth naturally than in women who have had a cesarean section, which may increase the risk of anal incontinence. Such result was similar to the research conclusions of Levin et al. [18]. It suggested that the AS thickness of primipara at 12 o'clock after vaginal delivery was thinner than the prenatal thickness, and there was no obvious difference in thickness in other directions. The measurement results of the puborectalis muscle revealed that there was no observable difference in the thickness of the bilateral puborectalis between vaginal delivery patients and cesarean section patients, showing no great difference, which may be related to the anterior and posterior diameter and area of the pelvic septum, which had to be studied and discussed in future clinical trials.

## 5. Conclusion

A freestyle KRR algorithm was constructed firstly, and GPU was adopted to optimize its computing time. Then, it was applied to 3D ultrasound images to analyze the injury of ASC of primiparas during vaginal delivery and cesarean section. It was found that the super 3D ultrasound images under the KRR algorithm could not only improve the diagnosis effect but also shorten the calculation time, improve the overall diagnosis efficiency, and can assist physicians in judging the injury of ASC of the primipara. The shortcomings of this study were that the number of selected patient samples was too small; the data led to a small scope of application of the research results and may also had some adverse effects on the results. In the process of follow-up research, it will consider increasing the sample of patients and expanding the scope of investigation. In addition, it will continue to study other factors affecting the injury of ASC and further explore new clinical treatment approaches for injury of ASC.

## Figures and Tables

**Figure 1:** Comparison on basic data of patients in two groups. (a–c) The age, weight and height, and birth weight, respectively.

**Figure 2:** Comparison on GPU acceleration effect of KRR algorithm. ^∗^Compared with other acceleration way, *P* < 0.05.

**Figure 3:** Comparison of CPU computing time under different kSize. ^∗^Compared with kSize = 10, *P* < 0.05; ^#^compared with kSize = 8, *P* < 0.05.

**Figure 4:** Comparison of computing time of multithreading CPU under different kSize. ^∗^Compared with kSize = 10, *P* < 0.05; ^#^compared with kSize = 8, *P* < 0.05.

**Figure 5:** Comparison of GPU computing time under different kSize. ^∗^Compared with kSize = 10, *P* < 0.05; ^#^compared with kSize = 8, *P* < 0.05.

**Figure 6:** The 3D tomographic images of AS of healthy people.

**Figure 7:** The 3D ultrasound image of the patient with defected AS.

**Figure 8:** The 3D ultrasound image of internal and external AS of a primipara (aged 26 years old).

**Figure 9:** Comparison of the measurement results of the proximal external AS between the two groups. ^∗^Compared with group B, *P* < 0.05.

**Figure 10:** Comparison of AS measurement results outside the anus in the two groups. ^∗^Compared with group B, *P* < 0.05.

**Figure 11:** Comparison of measurement results of distal external AS of the two groups of patients. ^∗^Compared with group B, *P* < 0.05.

**Figure 12:** Comparison of measurement results of distal internal AS of the two groups of patients. ^∗^Compared with group B, *P* < 0.05.

## Data Availability

The data used to support the findings of this study are available from the corresponding author upon request.
